# Targeting of CDKN1B by miR‐222‐3p may contribute to the development of intervertebral disc degeneration

**DOI:** 10.1002/2211-5463.12609

**Published:** 2019-03-12

**Authors:** Jianwei Liu, Jia Yu, Weiping Jiang, Maolin He, Jinmin Zhao

**Affiliations:** ^1^ Department of Osteology The Third Affiliated Hospital of Guangxi Medical University Nanning China; ^2^ Department of Spine Osteopathia The First Affiliated Hospital of Guangxi Medical University Nanning China; ^3^ Guangxi Key Laboratory of Regenerative Medicine International Joint Laboratory on Regeneration of Bone and Soft Tissue The First Affiliated Hospital of Guangxi Medical University Guangxi Medical University Nanning China

**Keywords:** CDKN1B, extracellular matrix, intervertebral disc degeneration, miR‐222‐3p, nucleus pulposus

## Abstract

MicroRNAs (miRNAs) are small endogenous non‐coding RNAs that can negatively regulate the expression of their complementary mRNA targets, and have been implicated in various pathophysiological processes. In this study, we examined the effect of miR‐222‐3p on intervertebral disc degeneration (IDD). We found that expression of miR‐222‐3p was significantly higher in IDD tissues than in normal intervertebral disc tissue, and report that overexpression of miR‐222‐3p remarkably increased apoptosis and reduced proliferation of nucleus pulposus (NP) cells. In addition, miR‐222‐3p promoted secretion of matrix metalloproteinase‐3, and decreased collagen type II and aggrecan production. Cyclin‐dependent kinase inhibitor 1B (CDKN1B) was identified as a direct target of negative regulation by miR‐222‐3p in NP cells, and expression of miR‐222‐3p was found to be negatively correlated with that of CDKN1B in IDD tissue. Finally, we observed that transfection with miR‐222‐3p dramatically reduced CDKN1B expression in NP cells. In conclusion, miR‐222‐3p may be involved in IDD development, possibly through targeting CDKN1B.

**Abbreviations**
3′‐UTR: 3′‐untranslated region
ACAN: aggrecan
CCK‐8: cell counting kit‐8
CDKN1B: cyclin‐dependent kinase inhibitor 1B
COL2A1: collagen type II
ECM: extracellular matrix
GAPDH: glyceraldehyde‐3‐phosphate dehydrogenase
GEO: gene expression omnibus
IDD: intervertebral disc degeneration
miRNA: microRNA
MMP‐3: matrix metalloproteinase‐3
MT: mutant
NP: nucleus pulposus
qRT‐PCR: quantitative real‐time PCR

Because of chronic low back pain and considerable economic expense, intervertebral disc degeneration (IDD) is a heavy load on society 1. Growing evidence has confirmed that gradual degeneration of the nucleus pulposus (NP) is responsible for the development of IDD, and the imbalance of extracellular matrix (ECM) breakdown and abnormal synthesis is a major cause of IDD 2, 3. NP cells are the most important cells of the intervertebral disc, and their aberrant activity is one of the leading cause of IDD 4. However, the pathological process of IDD and its potential mechanism remain unknown. Thus, finding specific targets on NP cells would help to better understand the development of IDD.

MicroRNAs (miRNAs) are small endogenous non‐coding RNAs. By binding to the 3′‐untranslated region (3′‐UTR) of the target mRNAs, miRNAs negatively regulate of the expression of complementary mRNA targets 5. miRNAs have been implicated in various cell pathophysiological processes, such as cell proliferation, apoptosis, and ECM metabolism. Accumulating evidence indicates that miRNAs are frequently dysregulated in the development of IDD. Although in recent years several miRNAs have come to be regarded as key players in the pathogenesis of IDD, the roles of many other miRNAs that are associated with pathogenesis of IDD remain to be elucidated

miR‐222‐3p has been implicated in several diseases, such as cancers 6, 7, 8, hypertrophic scar 9, and cardiovascular diseases 10; however, its role in IDD remains unclear. Cyclin‐dependent kinase inhibitor 1B (CDKN1B), also named p27kip1, has been reported to inhibit cell cycle progression G1–S transitions, and phosphorylation of CDKN1B at different sites altered its distribution in the nucleus and cytoplasm in different cancers 11, 12. *CDKN1B* was also a target gene of miR‐222‐3p in several cancers 13, 14, but the regulation by miR‐222‐3p of CDKN1B in NP cells remains unknown. Therefore, the aim of this study was to examine the effect and mechanism of miR‐222‐3p in IDD in targeting CDKN1B, and our results will provide a new therapeutic target for the treatment of IDD.

## Materials and methods

### Microarray data

The miRNA expression dataset of GSE19943 15 was downloaded from the Gene Expression Omnibus (GEO) database. This dataset has six samples, including three IDD NP tissues and three normal NP tissues. The microarray data were generated based on the GPL19446 platform (Exiqon human miRCURY LNA™ microRNA Array V11.0, Duesseldorf, Germany). The NP tissues in the normal group were grade I and in the IDD group grades IV and V by Pfirrmann grading 16.

### Collection of IDD tissue

The intervertebral disc tissues were collected from 30 IDD patients who underwent lumbar spine surgery from October 2017 to June 2018 in the Third Affiliated Hospital of Guangxi Medical University. IDD assessment was based on the criteria of Pfirrmann grading using MRI examination 16. Another 10 normal intervertebral disc tissues were obtained from patients who had traumatic lumbar fracture. The study protocols were approved by the ethics committee of Third Affiliated Hospital of Guangxi Medical University. All the procedures were in accordance with the World Medical Association Declaration of Helsinki Ethical Principles for Medical Research Involving Human Subjects, with signed written informed consent.

### NP cell isolation and culture

Human NP cells were obtained and cultured as previously described 17. The third passage of NP cells was used for further tests.

### miR‐222‐3p transfection

miR‐222‐3p mimic and inhibitors were chemically synthesized and purchased from GenePharma (Shanghai, China). Lipofectamine 2000 (Invitrogen, Carlsbad, CA, USA) was used for transaction as per the manufacturer's instructions. The NP cells were seeded at 1 × 10^5^ per well on 24‐well plates and then transfected with 80 ng plasmid, 5 ng *Renilla* luciferase vector pRL‐SV40, 50 nm miR‐222‐3p mimics and inhibitors by using Lipofectamine 2000. The final working concentration of miRNA was 100 nm. Experiments except the luciferase test were all conducted after 12 h of transfection.

### RNA extraction and quantitative real‐time PCR

RNA extraction and quantitative real‐time PCR (qRT‐PCR) were carried out using a general protocol of our laboratory 17. U6 and glyceraldehyde‐3‐phosphate dehydrogenase (*GAPDH*) were used as internal control for miR‐222‐3p and *CDKN1B*, respectively. The primer sequences of miR‐222‐3p, *CDKN1B*, U6 and *GAPDH* are listed in Table**** 1. The relative expression levels of miR‐222‐3p and *CDKN1B* were calculated using the 2^−ΔΔ*C*q^ method.

**Table 1:** Sequence of primers used in qRT‐PCR

Primer		Sequence (5′–3′)
miR‐222‐3p	Forward	5′‐AGC TAC ATC TGG CTA CTG G‐3′
	Reverse	5′‐GTA TCC AGT GCA GGG TCC‐3′
CDKN1B	Forward	5′‐AGT GTC TAA CGG GAG CCC TA‐3′
COL2A1	Reverse	5′‐AGT AGA ACT CGG GCA AGC TG‐3′
	Forward	5′‐TGA GCC ATG ATT CGC CTC G‐3′
	Reverse	5′‐CCC TTT GGT CCT GGT TGC C‐3′
ACAN	Forward	5′‐CTA CAC GCT ACA CCC TCG AC‐3′
	Reverse	5′‐ACG TCC TCA CAC CAG GAA AC‐3′
*MMP13*	Forward	5′‐CAC TCA CAG ACC TGA CTC GGT T‐3′
	Reverse	5′‐AAG CAG GAT CAC AGT TGG CTG G‐3′
U6	Forward	5′‐CTC GCT TCG GCA GCA CA‐3′
	Reverse	5′‐TGG TGT CGT GGA GTC G‐3′
GAPDH	Forward	5′‐GGC ACA GTC AAG GCT GAG AA TG‐3′
	Reverse	5′‐ATG GTG GTG AAG ACG CCA GTA‐3′

### Western blotting

Protein extraction and western blotting were performed according to the general protocol in our laboratory 18. Antibodies to CDKN1B (1 : 1000; Abcam, Cambridge, UK) and GAPDH (1: 2500; Abcam) were used as primary antibodies.

### Cell proliferation and apoptosis assay

Cell proliferation assay was conducted using a Cell Counting Kit‐8 (CCK‐8; Dojindo, Kumamoto, Japan) kit as instructed by the manufacturer. Cell apoptosis assays were quantified using an FITC Annexin V Apoptosis Detection Kit (Solarbio, Beijing, China) as previously described 17.

### Immunofluorescence microscopy

Cell immunofluorescence staining of collagen type II was observed and acquired using an epifluorescence microscope (Olympus BX53, Tokyo, Japan) equipped with a camera.

### Luciferase reporter assay

The binding site in the 3′‐UTR of *CDKN1B*, including *CDKN1B* wild‐type and *CDKN1B* mutant (MT) were cloned from human genomic DNA and then inserted into the KpnI and SacI sites of the pGL3 promoter vector (Realgene, Nanjing, China) in a dual‐luciferase reporter assay. After transfection for 48 h, the cells were collected and measured using a Dual‐Luciferase Assay Kit (Promega, Madison, WI, USA) according to the manufacturer's instructions.

### Statistical analysis

Data are shown as mean ± SD. Student's *t* test and one‐way ANOVA followed by Tukey's *post hoc* test were used to assess the statistical significance for numerical data (including the miR‐222‐3p expression in Table 2) using spss statistics v. 19.0 (IBM Corp., Armonk, NY, USA). Statistical significance was set at *P* < 0.05.

**Table 2:** Association of miR‐222‐3p expression with clinical parameters. Data are shown as mean ± SD. Student's *t* test was used to assess the statistical significance of miR‐222‐3p expression with age, gender and grade variables; one‐way ANOVA was used to assess the statistical significance miR‐222‐3p expression at the spine level

Variables	*n*	miR‐222‐3p expression	*P* value
Age			
< 50 years	18	7.52 ± 1.23	0.774
≥ 50 years	12	7.71 ± 1.46	
Gender			
Male	22	7.82 ± 1.58	0.787
Female	8	7.60 ± 1.37	
Grade			
IV	6	7.48 ± 1.21	0.031
V	24	7.92 ± 1.74	
Spine level			
L3/L4	8	7.62 ± 1.35	0.801
L4/L5	16	7.68 ± 1.39	
L5/S1	6	7.67 ± 1.38	

## Results

### miR‐222‐3p increased in IDD tissues

By analyzing the GSE19943 dataset, which included three IDD tissues and three normal intervertebral disc tissues, it was revealed that miR‐222‐3p was up‐regulated significantly in IDD tissues in contrast to normal intervertebral disc tissues (Fig. 1A, *P* < 0.05). In the clinical tissues, using the qRT‐PCR method, we found that the expression of miR‐222‐3p was greatly higher in IDD tissues than in normal intervertebral disc tissues as well (Fig. 1B, *P* < 0.01).

**Figure 1:** miR‐222‐3p expression in (A) the GSE19943 dataset and (B) the clinical tissues. Data are mean ± SD,* n* = 3, Student's *t* test was used to assess statistical significance: *P < 0.05, **P < 0.01.

### miR‐222‐3p correlated with IDD stage

Among the clinical intervertebral disc tissues, 10 intervertebral disc tissues in the normal group were grade I, and in the IDD group, six tissues were grade IV and 24 were grade V. No significant difference was detected between normal and IDD tissues with regard to age and gender (*P *>* *0.05). We then analyzed the miR‐222‐3p with the clinical parameters of IDD and found that miR‐222‐3p expression was up‐regulated in the advanced grade of IDD (*P *<* *0.05). There was no significant difference for age and gender in the IDD patients (*P *>* *0.05; Table 2.

### miR‐222‐3p suppresses NP cell proliferation and induces apoptosis

To examine the effect of miR‐222‐3p on the phenotype of NP cells, miR‐222‐3p mimics and inhibitors were transfected into NP cells. The expression of miR‐222‐3p was elevated significantly or decreased after transfecting using miR‐222‐3p mimics or inhibitors, respectively (Fig. 2A). The CCK‐8 assay showed that proliferation of NP cells was significant increased after transfecting miR‐222‐3p inhibitors (Fig. 2B), and flow cytometry showed that the apoptosis rate of NP cells was significantly reduced after transfecting with miR‐222‐3p inhibitors (Fig. 2C). Collectedly, reduction of miR‐222‐3p was able to facilitate proliferation and suppress apoptosis of NP cells.

**Figure 2:** miR‐222‐3p affects the phenotype of NP cells. (A) miR‐222‐3p expression in NP cells after transfecting with miR‐222‐3p mimics and inhibitors. (B) NP cell proliferation rate after transfecting with miR‐222‐3p mimics and inhibitors. (C) NP cell apoptosis rate after transfecting with miR‐222‐3p mimics and inhibitors. Mean ± SD,* n* = 3; one‐way ANOVA followed by Tukey's *post hoc* test was used to assess statistical significance: *P < 0.05, **P < 0.01.

### miR‐222‐3p inhibited ECM production of NP cells

Collagen type II (COL2A1) and aggrecan (ACAN) are common cytokines used to characterize ECM production in NP cells, whereas MMP‐3 suppresses ECM synthesis 19, 20. In this study, when the miR‐222‐3p mimics and inhibitors were transfected into NP cells, we observed that the mRNA and protein level of COL2A1 and ACAN were decreased with miR‐222‐3p overexpression, while the mRNA and protein expression of MMP‐3 was increased with overexpression of miR‐222‐3p (Fig. 3A–C). In addition, the immunostaining also indicated that miR‐222‐3p could reduce COL2A1 expression (Fig. 3D). All these results demonstrated that miR‐222‐3p uptake can reduce the activity and production of ECM in NP cells.

**Figure 3:** Expression of COL2A1, ACAN and MMP‐3 after transfecting with miR‐222‐3p. (A) Expression of COL2A1, ACAN and MMP‐3 mRNA after transfecting with miR‐222‐3p. (B) Western blot images of COL2A1, ACAN and MMP‐3 protein after transfecting with miR‐222‐3p. (C) Expression of COL2A1, ACAN and MMP‐3 protein after transfecting with miR‐222‐3p. (D) Immunostaining images of COL2A1 after transfecting with miR‐222‐3p; scale bar: 100 μm. Mean ± SD,* n* = 3; one‐way ANOVA followed by Tukey's *post hoc* test was used to assess statistical significance: *P < 0.05, **P < 0.01.

### Luciferase reporter assay confirmed that miR‐222‐3p directly targeted CDKN1B

Three miRNA target gene databases (Targetscan, http://www.targetscan.org/mamm_31/) revealed that the miR‐222‐3p sequence has four binding sites for the 3′‐UTR of *CDKN1B*, suggesting that *CDKN1B* may be a potential target gene of miR‐222‐3p (Fig. 4A). Then, through using the dual‐luciferase reporter assay, we found that miR‐222‐3p overexpression significantly reduced the relative luciferase activity of the reporter gene for wild‐type, but not mutant *CDKN1B* in NP cells (Fig. 4B), indicating that miR‐222‐3p directly targeted the 3′‐UTR of *CDKN1B* in NP cells.

**Figure 4:** Cyclin‐dependent kinase inhibitor 1B was a direct target of miR‐222‐3p. (A) Targetscan database showed that miR‐222‐3p sequence has four binding sites for the 3′‐UTR of CDKN1B. (B) Luciferase reporter assay showed that miR‐222‐3p significantly reduced the luciferase activity of wild‐type, but not mutant *CDKN1B* in NP cells. Mean ± SD,* n* = 3; one‐way ANOVA followed by Tukey's *post hoc* test was used to assess statistical significance: *P < 0.05, **P < 0.01.

### miR‐222‐3p negatively correlated with CDKN1B and reduced its expression

Using qRT‐PCR method to measure the CDKN1B expression in IDD tissue, we observed a negatively correlated expression of miR‐222‐3p to CDKN1B (Fig. 5A). We then transfected NP cells with miR‐222‐3p mimics and inhibitor for 24 h and measured the CDKN1B mRNA and protein in NP cells. The results indicated that CDKN1B mRNA and protein were significantly decreased after miR‐222‐3p mimic transfection (Fig. 5B–D), indicating that miR‐222‐3p targeted and negatively regulates CDKN1B at the post‐transcriptional level in NP cells.

**Figure 5:** Association of miR‐222‐3p with CDKN1B. (A) Correlation analysis of miR‐222‐3p and CDKN1B in IDD tissue. (B) Expression of CDKN1B mRNA in NP cells after transfecting with miR‐222‐3p. (C) Expression of CDKN1B protein in NP cells after transfecting with miR‐222‐3p. (D) Western blot images of CDKN1B protein after transfecting with miR‐222‐3p. Mean ± SD,* n* = 3; one‐way ANOVA followed by Tukey's *post hoc* test was used to assess the statistical significance: *P < 0.05, **P < 0.01.

## Discussion

In this study, we measured the miRNAs in the GSE19943 dataset and clinical specimens using the qRT‐PCR method. The results indicated that miR‐222‐3p was dramatically increased in IDD tissue compared with normal intervertebral disc. In addition, our results also indicated that expression of miR‐222‐3p was much higher in the advance grade of IDD compared with that in early grade, suggesting miR‐222‐3p is involved in the pathogenesis of IDD. We next examined the effect on the change of NP cell phenotype and observed that down‐regulation of miR‐222‐3p could suppress NP cells apoptosis and induce proliferation, that it subsequently reduced the production of COL2A1 and ACAN, and that it increased the MMP‐3 expression in NP cells. Our results demonstrated that *CDKN1B* is a direct targeted gene of miR‐222‐3p in NP cells, and CDKN1B was negatively correlated with miR‐222‐3p in IDD tissue.

miR‐222‐3p expression was reported to be enhanced in breast cancer 21, gastric cancer 22, and lung cancer 23; however, lower miR‐222‐3p levels were observed in severe myocardial fibrosis as compared to non‐severe fibrosis 24. Thus, the expression of miR‐222‐3p is varied in different diseases. With regard to the effect of miR‐222‐3p on cells, several studies have observed that miR‐222‐3p was associated with the proliferation, apoptosis, invasion and migration of some cancer cells 6, 25. Studies also showed that miR‐222‐3p is involved in regulation of mitochondrial dysfunction in response to transmissible gastroenteritis virus infection 26 and erythroid differentiation 27. Our results showed that down‐regulation of miR‐222‐3p could greatly inhibit apoptosis and enhance proliferation of NP cells, indicating that miR‐222‐3p expression was closely correlated with the NP cell phenotype.

In the current study, we also detected the expression of COL2A1, ACAN and MMP‐3 after NP cells were transfected by miR‐222‐3p mimics and inhibitors. It is well known that the progressive loss of ECM is a hallmark of IDD, while MMP‐3 is the main enzymes that degrades collagen II and expression of MMP‐3 was increased in IDD tissue compared with healthy controls 19, 20. Moreover, other research reported that miR‐222‐3p was associated with ECM production in axial spondyloarthritis 28. In agreement with the results for the phenotypic changes of NP cells, we observed that miR‐222‐3p overexpression significantly down‐regulated the expression of COL2A1 and ACAN mRNA and protein levels, and up‐regulated the MMP‐3 mRNA and protein levels in NP cells. All in all, miR‐222‐3p will modulate the development of IDD through inhibiting the activity of NP cells.

Evidence has shown that miR‐222‐3p could target several genes, and a relationship of miR‐222‐3p‐targeted *CDKN1B* has been implicated in breast cancer cells 29 and vascular smooth muscle cells 30, but this relationship has not been reported in NP cells. CDKN1B has high expression in nearly all the tissue of the body, and is involved in several forms of cell growth regulation including cell cycle, apoptosis, and phenotype expression 31. The role of CDKN1B is influenced mainly by two mechanisms: the level of transcription and protein stability, and its subcellular localization 32. Our work confirmed that miR‐222‐3p directly targeted CDKN1B in NP cells, and negatively regulated the CDKN1B level, which was also correlated to IDD. Therefore, this indicates that miR‐222‐3p targets CDKN1B then regulates IDD progression.

## Conclusion

In this paper, our results revealed that miR‐222‐3p was significantly increased in IDD tissues and associated with IDD grade. Furthermore, CDKN1B was demonstrated to be the potential target of miR‐222‐3p, which facilitates IDD development. Our results provide a potential theory of IDD development, and a potential target for the treatment of IDD.

## Conflict of interest

The authors declare no conflict of interest.

## Author contributions

Study concept and design: JWL, WPJ, MLH and JMZ. Performance of the experiments: JWL and JY. Data analysis and interpretation: JWL, JY and WPJ. Manuscript writing and review: JWL, JY and WPJ. All authors read and approved the final manuscript.

## References

[1] Millward‐Sadler SJ , Costello PW , Freemont AJ and Hoyland JA (2009) Regulation of catabolic gene expression in normal and degenerate human intervertebral disc cells: implications for the pathogenesis of intervertebral disc degeneration. Arthritis Res Ther 11, R65.1943550610.1186/ar2693PMC2714110

[2] Wang SZ , Rui YF , Lu J and Wang C (2014) Cell and molecular biology of intervertebral disc degeneration: current understanding and implications for potential therapeutic strategies. Cell Prolif 47, 381–390.2511247210.1111/cpr.12121PMC6495969

[3] Zhu Y , Tan J , Zhu H , Lin G , Yin F , Wang L , Song K , Wang Y , Zhou G and Yi W (2017) Development of kartogenin‐conjugated chitosan‐hyaluronic acid hydrogel for nucleus pulposus regeneration. Biomater Sci 5, 784–791.2826173310.1039/c7bm00001d

[4] Gan Y , Li P , Wang L , Mo X , Song L , Xu Y , Zhao C , Ouyang B , Tu B , Luo L *et al* (2017) An interpenetrating network‐strengthened and toughened hydrogel that supports cell‐based nucleus pulposus regeneration. Biomaterials 136, 12–28.2850559710.1016/j.biomaterials.2017.05.017

[5] Engels BM and Hutvagner G (2006) Principles and effects of microRNA‐mediated post‐transcriptional gene regulation. Oncogene 25, 6163–6169.1702859510.1038/sj.onc.1209909

[6] Gong L , Zhang W , Yuan Y , Xing X , Li H and Zhao G (2018) miR‐222 promotes invasion and migration of ovarian carcinoma by targeting PTEN. Oncol Lett 16, 984–990.2996317310.3892/ol.2018.8743PMC6019905

[7] Sun Q , Jiang CW , Tan ZH , Hou LY , Dong H , Liu K , Sun G , Liu YJ , Wang YQ , Lu XC *et al* (2017) MiR‐222 promotes proliferation, migration and invasion of lung adenocarcinoma cells by targeting ETS1. Eur Rev Med Pharmacol Sci 21, 2385–2391.28617551

[8] Wei F , Ma C , Zhou T , Dong X , Luo Q , Geng L , Ding L , Zhang Y , Zhang L , Li N *et al* (2017) Exosomes derived from gemcitabine‐resistant cells transfer malignant phenotypic traits via delivery of miRNA‐222‐3p. Mol Cancer 16, 132.2874328010.1186/s12943-017-0694-8PMC5526308

[9] Zhang Y , Zhang L , Zhang Q , Hong W and Lin X (2017) microRNA‐222 regulates proliferation and apoptosis of fibroblasts in hypertrophic scar via matrix metalloproteinase 1. Zhejiang Da Xue Xue Bao Yi Xue Ban 46, 609–617.2965866310.3785/j.issn.1008-9292.2017.12.06PMC10396847

[10] Ding S , Huang H , Xu Y , Zhu H and Zhong C (2017) MiR‐222 in cardiovascular diseases: physiology and pathology. Biomed Res Int 2017, 4962426.2812755710.1155/2017/4962426PMC5239839

[11] Hnit SS , Xie C , Yao M , Holst J , Bensoussan A , De Souza P , Li Z and Dong Q (2015) p27(Kip1) signaling: Transcriptional and post‐translational regulation. Int J Biochem Cell Biol 68, 9–14.2627914410.1016/j.biocel.2015.08.005

[12] Whitcomb EA , Tsai YC , Basappa J , Liu K , Le Feuvre AK , Weissman AM and Taylor A (2018) Stabilization of p27(Kip1)/CDKN1B by UBCH7/UBE2L3 catalyzed ubiquitinylation: a new paradigm in cell‐cycle control. FASEB J 33, 1235–1247.3011388210.1096/fj.201800960RPMC6355086

[13] Sun C , Li N , Zhou B , Yang Z , Ding D , Weng D , Meng L , Wang S , Zhou J , Ma D *et al* (2013) miR‐222 is upregulated in epithelial ovarian cancer and promotes cell proliferation by downregulating P27(kip1.). Oncol Lett 6, 507–512.2413735610.3892/ol.2013.1393PMC3789083

[14] Wang C , Wang WJ , Yan YG , Xiang YX , Zhang J , Tang ZH and Jiang ZS (2015) MicroRNAs: New players in intervertebral disc degeneration. Clin Chim Acta 450, 333–341.2636826610.1016/j.cca.2015.09.011

[15] Wang HQ , Yu XD , Liu ZH , Cheng X , Samartzis D , Jia LT , Wu SX , Huang J , Chen J and Luo ZJ (2011) Deregulated miR‐155 promotes Fas‐mediated apoptosis in human intervertebral disc degeneration by targeting FADD and caspase‐3. J Pathol 225, 232–242.2170648010.1002/path.2931

[16] Pfirrmann CW , Metzdorf A , Zanetti M , Hodler J and Boos N (2001) Magnetic resonance classification of lumbar intervertebral disc degeneration. Spine (Phila Pa 1976) 26, 1873–1878.1156869710.1097/00007632-200109010-00011

[17] Liu J , Jiang T , He M , Fang D , Shen C , Le Y , He M , Zhao J and Zheng L (2018) Andrographolide prevents human nucleus pulposus cells against degeneration by inhibiting the NF‐kappaB pathway. J Cell Physiol 234, 9631–9639.3037069410.1002/jcp.27650

[18] Jiang T , Zhou B , Huang L , Wu H , Huang J , Liang T , Liu H , Zheng L and Zhao J (2015) Andrographolide exerts pro‐osteogenic effect by activation of Wnt/beta‐catenin signaling pathway in vitro. Cell Physiol Biochem 36, 2327–2339.2627943710.1159/000430196

[19] Wang X , Wang H , Yang H , Li J , Cai Q , Shapiro IM and Risbud MV (2014) Tumor necrosis factor‐alpha‐ and interleukin‐1beta‐dependent matrix metalloproteinase‐3 expression in nucleus pulposus cells requires cooperative signaling via syndecan 4 and mitogen‐activated protein kinase‐NF‐kappaB axis: implications in inflammatory disc disease. Am J Pathol 184, 2560–2572.2506353010.1016/j.ajpath.2014.06.006PMC4188173

[20] Wang H , Hao P , Zhang H , Xu C and Zhao J (2018) MicroRNA‐223 inhibits lipopolysaccharide‐induced inflammatory response by directly targeting Irak1 in the nucleus pulposus cells of intervertebral disc. IUBMB Life 70, 479–490.2970787810.1002/iub.1747

[21] Amini S , Abak A , Estiar MA , Montazeri V , Abhari A and Sakhinia E (2018) Expression analysis of MicroRNA‐222 in breast cancer. Clin Lab 64, 491–496.2973909010.7754/Clin.Lab.2017.171002

[22] Tan X , Tang H , Bi J , Li N and Jia Y (2018) MicroRNA‐222‐3p associated with Helicobacter pylori targets HIPK2 to promote cell proliferation, invasion, and inhibits apoptosis in gastric cancer. J Cell Biochem 119, 5153–5162.2922753610.1002/jcb.26542

[23] Di Fazio P , Maass M , Roth S , Meyer C , Grups J , Rexin P , Bartsch DK and Kirschbaum A (2017) Expression of hsa‐let‐7b‐5p, hsa‐let‐7f‐5p, and hsa‐miR‐222‐3p and their putative targets HMGA2 and CDKN1B in typical and atypical carcinoid tumors of the lung. Tumour Biol 39, 1010428317728417.2901739310.1177/1010428317728417

[24] Verjans R , Peters T , Beaumont FJ , van Leeuwen R , van Herwaarden T , Verhesen W , Munts C , Bijnen M , Henkens M , Diez J *et al* (2018) MicroRNA‐221/222 family counteracts myocardial fibrosis in pressure overload‐induced heart failure. Hypertension 71, 280–288.2925507310.1161/HYPERTENSIONAHA.117.10094

[25] Chu YW , Wang CR , Weng FB , Yan ZJ and Wang C (2018) MicroRNA‐222 contributed to cell proliferation, invasion and migration via regulating YWHAG in osteosarcoma. Eur Rev Med Pharmacol Sci 22, 2588–2597.2977144210.26355/eurrev_201805_14952

[26] Zhao X , Song X , Bai X , Tan Z , Ma X , Guo J , Zhang Z , Du Q , Huang Y and Tong D (2018) microRNA‐222 attenuates mitochondrial dysfunction during transmissible gastroenteritis virus infection. Mol Cell Proteomics 18, 51–64.3025787810.1074/mcp.RA118.000808PMC6317483

[27] Jiang L , Wang X , Wang Y and Chen X (2018) Quantitative proteomics reveals that miR‐222 inhibits erythroid differentiation by targeting BLVRA and CRKL. Cell Biochem Funct 36, 95–105.2936833810.1002/cbf.3321

[28] Prajzlerova K , Grobelna K , Husakova M , Forejtova S , Jungel A , Gay S , Vencovsky J , Pavelka K , Senolt L and Filkova M (2017) Association between circulating miRNAs and spinal involvement in patients with axial spondyloarthritis. PLoS ONE 12, e0185323.2893800610.1371/journal.pone.0185323PMC5609864

[29] Wang DD , Yang SJ , Chen X , Shen HY , Luo LJ , Zhang XH , Zhong SL , Zhao JH and Tang JH (2016) miR‐222 induces Adriamycin resistance in breast cancer through PTEN/Akt/p27(kip1) pathway. Tumour Biol 37, 15315–15324.2769966510.1007/s13277-016-5341-2

[30] Xu Y , Bei Y , Shen S , Zhang J , Lu Y , Xiao J and Li X (2017) MicroRNA‐222 promotes the proliferation of pulmonary arterial smooth muscle cells by targeting P27 and TIMP3. Cell Physiol Biochem 43, 282–292.2885442810.1159/000480371

[31] Abbastabar M , Kheyrollah M , Azizian K , Bagherlou N , Tehrani SS , Maniati M and Karimian A (2018) Multiple functions of p27 in cell cycle, apoptosis, epigenetic modification and transcriptional regulation for the control of cell growth: a double‐edged sword protein. DNA Repair (Amst) 69, 63–72.3007537210.1016/j.dnarep.2018.07.008

[32] le Sage C , Nagel R and Agami R (2007) Diverse ways to control p27Kip1 function: miRNAs come into play. Cell Cycle 6, 2742–2749.1798686510.4161/cc.6.22.4900

